The article "Analysis of the Relationship between Transformational Leadership and Educational Management in Higher Education Based on Deep Learning" was published in 2022. Journal: Comput Intell Neurosci.

# Analysis of the Relationship between Transformational Leadership and Educational Management in Higher Education Based on Deep Learning

**DOI:** 10.1155/2022/5287922

**Published:** 2022-06-15

**Authors:** Haiying Meng

**Affiliations:** School of Business Sanda University, Shanghai 201209, China

## Abstract

Leadership behavior has been emphasized as one of the most important influencing factors in the innovation process. Leaders can encourage subordinates to innovate by creating the right environment, promoting knowledge integration, and setting specific goals. However, different leadership styles make different decisions and behaviors in the innovation process, and the final innovation effect is also different. Today, in the context of China, most business leaders still adopt “paternalistic” or “authoritarian” leadership behaviors, but more and more entrepreneurs and scholars are aware of the importance of this leadership style in enhancing employee creativity. Authoritarian leaders are more likely to exercise more control and supervision over team members, limit the autonomy of team members, and reduce work initiative and creativity. Although the positive effect of transformational leadership on employee creativity has been recognized by some scholars, in the real work environment, this leadership style rarely appears, especially in the context of China. This study first constructs a theoretical model of how transformational leaders in colleges and universities affect educational management innovation through the atmosphere of school organizational innovation, based on the deep learning theory and other related research results, and then puts forward research hypotheses on this basis. Secondly, a measurement scale was designed according to the existing research results, and the scale was revised through the pretest to form the formal questionnaire of this study. This research uses cluster sampling and random sampling to conduct a questionnaire survey on 1022 college teachers and uses the SPSS20.0 and AMOS21.0 to conduct an empirical analysis on the survey data. Each measurement scale was tested by exploratory factor analysis and confirmatory factor analysis. The experimental results show that the transformational leadership style of college principals has a positive impact on teachers' teaching innovation. There is a positive correlation between the influence of charisma and teachers' teaching management, and there is a positive correlation between intellectual stimulation and teachers' teaching management.

## 1. Introduction

The rapid growth and increasing globalization of technology have brought complex challenges and significant changes to higher education institutions since the twenty-first century; Basham, for colleges and universities, effectively solves problems and makes full use available resources. Therefore, there is a huge demand for new definitions and approaches to the leadership and management of higher education institutions. Leaders are expected to work more effectively in rapidly changing environments and to respond appropriately to these challenges. To facilitate change, leaders must respect each other's knowledge and find new ways to identify and solve complex problems and challenges. Since James McGregor Burns first conceptualized leadership as transactional or transformational leadership in 1978, transformational leadership has quickly become the choice for a large number of studies and applications of leadership theory. A wealth of evidence has accumulated to demonstrate the effectiveness of transformational leaders in a variety of settings around the world. Much of the leadership literature asserts the positive effects of transformational leadership on followers. In addition, numerous studies have shown that transformational leadership has a profoundly beneficial impact on the achievement of organizational goals. In higher education, academics have spent years studying the needs, multiple roles, and criticality of organizational leaders. Research shows that leadership styles at all levels of higher education institutions are complex and multidimensional. This research focuses on uncovering how transformational leadership is applied in higher education management settings. Specifically, two research questions are mainly discussed: (1) Is transformational leadership considered to be effective leadership in an academic setting? (2) How does transformational leadership affect performance? By exploring the hypothesis of the relationship between various related variables between transformational leadership and educational management, it is expected to provide corresponding inspiration based on the analysis results and the current situation of educational management development [1–9].

## 2. Related Work

After entering the 1970s, leadership theory was influenced by various academic thoughts, such as business leadership theories, new philosophies, and social thoughts, which led to the emergence of new leadership theories such as transactional, transformational, charismatic, and ethical leadership. Among them, the most influential and most respected leadership theory in management practice is the transformational leadership proposed by Burns. Over the past few decades, many researchers have studied transformational leadership and performance in a variety of settings. In higher education, several scholars have explored the effectiveness of transformational leadership in relation to the president. Others surveyed middle-level transformational leaders, including department chairs and deans. Basham focuses on the characteristics and traits of college presidents who are considered transformational leaders in America. His research supports the published and perceived characteristics of higher education leaders and their approaches to changing the learning climate in their organizations. The research highlights the group and individual qualities needed to create a transformative environment that fosters transformational leadership. Mattar aims to explore whether the characteristics and leadership styles of effective university leaders in Lebanon match those of transformational leaders. The results show that an effective leader largely accounts for most of the traits and attitudes that define transformational leaders. A transformational leader inspires and motivates all employees on campus, including faculty and staff, by fostering the spirit of co-workers, creating a friendly work environment, and respecting teamwork. On the other hand, the leadership styles of middle managers and their relationship with leader effectiveness were studied in different cultural contexts. Jones and Rudd found similar results that transformational leadership behaviors were used more often by the most effective and successful leaders, followed by transactional leadership and less laissez-faire leadership. Pixi et al. sought to find out whether the characteristics and leadership styles of effective heads of academic departments in Malaysian universities are related to transformational leadership. In their study, inspirational motivation and idealized influence received the highest average scores, while intellectual stimulation and personalized consideration received the lowest average scores. The findings also suggest that, as a dimension of transactional leadership, contingent rewards have a significant impact on leadership effectiveness. These findings are consistent with many previous studies. Leaders' scores on the MLQ's Transformational Leadership Scale correlated significantly with measures of leader effectiveness. Furthermore, contingent rewards are often closely related to a leader's effectiveness. Existing studies have shown that transformational and transactional leadership theories have always been hotspots in management and school management research fields, and there have been relatively abundant studies on theoretical overview and dimensional structure. However, in the field of schools, transformational leadership mostly focuses on the influence of the principal's leadership style on teachers' psychological motivation and sense of efficacy and is limited to the single leadership style of transformational leadership. Based on the existing research, this research will focus on sorting out the role of transformational leadership in the atmosphere of school organization and teaching management, discussing their impact on teachers' teaching management, and exploring the mechanism of action between variables. Comparative analysis is beneficial to teachers' teaching [10–15].

## 3. Study Design

### 3.1. Conceptual Model

This study proposes a research framework for university leadership, school organizational innovation, and teacher teaching management. The principal's leadership is the independent variable, the teachers' teaching management is the dependent variable, and the school's organizational management climate is the mediating variable. Referring to Bass's classic literature, it can be seen that leadership effectiveness, organizational philosophy, team operation, learning growth, working conditions, environmental atmosphere, educational value, and policy are the main measures of college leadership management. Dimensions are more of a measure of transformational leadership, including leadership effectiveness, organizational philosophy, team operation, learning and growth, working conditions, environmental atmosphere, and the seven dimensions of educational value and policy. According to Chen Shuangcai, Wang Zhenhong, and You Xuqun's related research studies, teachers' teaching management is divided into five dimensions: conceptual thinking management, teaching content management, teaching method management, teaching resource management, and multievaluation management [16].

### 3.2. Research Hypothesis

There has been extensive and rich research in the corporate field on the impact of leadership styles on subordinates' innovative behavior. Among the many factors that affect the innovation performance of organizational members, the behavior of leaders is considered to be the primary condition for introducing innovative ideas, promoting organizational change, setting innovation performance goals, and providing members with innovative resources, which can create a sustainable innovation environment for organizational members. Summarizing existing research, the principal's leadership style has an important impact on the school organization. Effective leadership not only pays attention to the realization of organizational goals but also pays attention to the overall cohesion of the school, the individual development of teachers, and their satisfaction with their work. Teachers demonstrate organizational goals and provide a rich teaching resource environment and a reasonable innovation mechanism. School leaders with transformational leadership have a positive role in guiding the innovation of the entire organization. Existing theories widely believe that transformational leadership has a more positive impact on organizational innovation than transactional leadership. Second, transformational leadership supports innovative learning processes in the organization and focuses on building mutual trust with teachers. The principal pursues organizational reform and innovation by taking himself as an example and fully encourages active and adventurous reform behaviors, thereby stimulating teachers' active exploration of teaching methods and teaching content and constantly seeking new and changing learning. The environment leads teachers to achieve the shared vision of the school. Based on the above analysis, we propose the following assumptions:

  H1: the transformational leadership of college principals has a positive impact on teachers' teaching management
  H1a: there is a positive correlation between charisma influence and teacher teaching management
  H1b: there is a positive correlation between vision motivation and teacher teaching management
  H1c: there is a positive correlation between individualized care and teacher teaching management
  H1d: there is a positive correlation between intellectual stimulation and teacher teaching management

### 3.3. Research Tools

The part of measuring transformational leadership style in the Multifactor Leadership Questionnaire (Form5X) compiled by Bass was used, which was later revised by domestic scholar Li Chaoping. This article adopts the domestic revision, in which the transformational leadership style has four dimensions: charismatic influence, individualized care, intellectual stimulation, and vision stimulation. This study follows Bass's multifactor leadership style questionnaire to measure transactional leadership, including contingency rewards, active exception management, and passive exception management. The scale includes 35 items, measured on a 5-point scale (from 5 = completely agree to 1 = completely disagree) [17–19]. The details are shown in Table 1.

### 3.4. Data Collection Methods

The main research object of this research is college teachers. A total of 300 teachers from colleges and universities in the survey area were randomly selected to fill in the questionnaire as the survey sample for the test; a formal questionnaire survey was conducted. First, select 30 colleges and universities in the H region by the cluster sampling method, and then select 100 teachers from each school by the random sampling method. Teachers' personal information includes teachers' gender, teaching age, education background, job title, professional title, teaching period, and teaching subject. It mainly focuses on the school's leadership style perceived by teachers, the school's innovative atmosphere, and the level of teaching innovation they have [20].

## 4. Empirical Research

### 4.1. Reliability and Validity Test

To test the validity and reliability of the scale, the reliability test of the formal questionnaire still uses the Cronbach alpha coefficient. According to Bryman et al. (1997), if the internal reliability *α* coefficient is above 0.8, it means that the scale has high reliability; if the reliability of the prepared research tool is below 0.6, the measurement tool needs to be recompiled.  Table 2 shows the reliability analysis of the formal questionnaire.

The above reliability test results show that the Cronbach *α* coefficients of transformational leadership, transactional leadership, school organizational innovation atmosphere, teacher teaching innovation scale, and subdimensions are all above 0.7, indicating that the reliability level of the scale is high. Each measurement item has a high internal consistency, which enables further analysis of the data.

### 4.2. Validity Test

According to the previous validity analysis results, the measurement tools used are mature scales that have been widely used and modified, indicating that the questionnaire has high content validity after factor analysis and principal component analysis (principal component analysis) to obtain the optimal factor structure of the scale, which ensures the construct validity of the scale. At this point, all factors and items of the scale have been determined. What needs to be explored is whether the factor structure model of the scale is consistent with the actual search data and whether the index variable can be effectively used as the measurement variable of the factor construct. The factor analysis procedure is confirmatory factor analysis (referred to as CFA). In this study, seven goodness-of-fit indicators (*X*^2^/d*f*, RMR, GFI, IFI, CFI, TLI, and RMSEA) were used to evaluate the model fit.

1. The chi-square degree of freedom ratio *X*^2^/d*f* can be used as an indicator of whether the model fits. The smaller the value is, the better the covariance matrix of the model fits the observed data. The chi-squared degrees of freedom ratios between 1 and 5 indicate an acceptable fit of the hypothesized model to the sample data.
2. The residual mean square and square root RMR refer to the difference between the variance-covariance matrix of the measured data and the variance-covariance matrix implied by the theoretical model. According to Qiu Haozheng, when the RMR value is below 0.05, it is an acceptable fit model.
3. The fitness index GFI is used to represent the ratio of “the sum of the squares of the difference between the observation matrix of the sample data and the theoretically constructed replication matrix” and the “observed variance.” When the GFI value is greater than 0.9, it represents the actual data and model path map has a good fit.
4. The value of the modified fitting index IFI and the modified fitting index CFI is between 0 and 1. The closer to 1, the better the fit of the model, which is generally used to judge whether the model path map is suitable for the actual data. The standard is above 0.9.
5. The nonregular fit index TLI is used to compare the degree of fit between two opposing models. The data of this index is between 0 and 1, and the standard or critical value of general fit is also above 0.9.
6. The asymptotic residual mean square and square root RMSEA is an absolute value indicator that does not require a baseline model. Steiger (1989) believes that when the RMSEA value is less than 0.05, it means that the model has a high degree of fitness. The details are shown in Table 3.

Confirmatory factor analysis on transformational leadership and its four dimensions found that among the evaluation indicators of the overall model goodness of fit, the chi-square degree of freedom *x*^2^/d*f* ratio was less than 3, the fitness index GFI was greater than 0.9, and the progressive residual mean square and square root RMSEA were less than 0.08, and the other indicators all met the discriminant criteria. It can be seen that the overall model has good goodness of fit, and the model chart hypothesis of the scale's confirmatory factor analysis is statistically supported. The details are shown in Figure 1.

### 4.3. Descriptive Statistics of the Data

Before conducting formal data analysis, in order to ensure the accuracy of data analysis, the discrete level and concentration degree of the variables of transformational leadership, transactional leadership, school organizational innovation, and teachers' teaching innovation variables were analyzed first, that is, the average of each variable (Mean) and standard deviation (Std. deviation), which improves the validity of data analysis results to a certain extent, but simply comparing the mean of each variable does not indicate that the difference has reached a statistically significant level, and a dependent sample variance analysis at each level is required.

The results of descriptive statistics and dependent sample variance analysis of the Transformational Leadership Scale show that the overall test of the mean difference of the four dimensions has reached a significant level, and the post hoc test shows that the average score of charisma is significantly higher than the average of the other three dimensions. The average score of individualized care is significantly lower than the average score of the other three dimensions. It can be considered that the teacher's perception of the principal's personal concern for himself is the least, and the feeling of the influence of charm is the strongest. At the same time, the standard deviation of each variable is less than 1, indicating that the level of the sample data set is relatively high. The details are shown in Table 4.

### 4.4. Regression Analysis considering the Influence of Control Variables

When two variables are significantly correlated, correlation analysis can only reflect the degree and direction of the correlation between the two variables. Regression analysis is based on the linear relationship between variables, further predicts the causal relationship between two variables, and uses an independent variable to predict the situation of the calibration variable. Under the premise of controlling for background variables such as gender and age of teachers, this study uses the principal's transformational leadership and transactional leadership as predictors to test the regression relationship between teachers' teaching innovation and the school standard variable and uses the stepwise multiple regression analysis method (Stepwise) to test the mediating effect of the school's organizational innovation climate. In the process of using multiple regression analysis, it is necessary to pay attention to whether there is a collinearity problem between the variables, that is, the correlation between the independent variables is too high, which will interfere with the fitting of the regression model. In order to test whether there is collinearity between independent variables, this study uses three indicators: tolerance (Tolerance), variance inflation factor (VIF), and serial correlation (Durbin–Watson).

#### 4.4.1. Collinearity Diagnosis

1. Tolerance: tolerance is equal to (1-*R*2), where *R*2 represents the square of the multivariate correlation coefficient between independent variables. The value range of tolerance is between 0 and 1. If the tolerance of an independent variable is too small, it means that there is a collinearity problem between the variable and other independent variables; if the value is close to 0, it means that this variable is almost a linear combination of other variables. The estimated value of the regression coefficient of the variable is not stable enough, and the calculated value of the regression coefficient will also have a large error.
2. Variance inflation factor: the variance inflation factor (VIF) is the reciprocal of tolerance, which reflects the possible common change trend between independent variables. If there is a high correlation, it means that the distortion of the regression model is more serious. Usually, the larger the value of VIF, the smaller the tolerance between independent variables and the more likely there is a collinearity problem. When the VIF value in the regression model is greater than 0 and less than 10, it can be considered that there is no multicollinearity between independent variables; if it is greater than 10, it means that the multicollinearity between independent variables is serious.
3. Sequence correlation: sequence correlation (Durbin–Watson) is a kind of correlation that exists in the regression model, that is, the significant correlation between different sample points. Serial correlation can be found by computing the Durbin–Watson value in the regression model, which can range from 0 to 4. When DW = 0, it means that there is a positive correlation between the residual values; when the value approaches 2, it means that there is no correlation between the residual items; when the DW value tends to 4, it means there is no serial correlation between them.

#### 4.4.2. Regression Analysis between Variables

The details are shown in Table 5. Firstly, under the premise of controlling demographic variables such as teacher gender, teaching age, education background, and teaching subject, transformational leadership was introduced into the first-level regression model, and the Durbin–Watson value of the serial correlation was 1.881, ranging from 0 to 1.4, indicating that there is no autocorrelation in the model. The tolerance value is between 0.454 and 0.978, the maximum value of the variance inflation factor VIF is 2.203, and there is no serious collinearity in the model. Its multivariate correlation coefficient *R* value is 0.621, the coefficient of determination *R*2 value is 0.386, the adjusted *R* square value is equal to 0.381, and the estimated standard error is 9.272, so transformational leadership can explain 38.6% of the total variance of teacher teaching innovation in the dependent variable. The standardized regression coefficient *β* value is 0.615, which shows that transformational leadership has a significant positive impact on teachers' teaching innovation and that transformational leadership has a positive predictive effect on teachers' teaching innovation as a whole. Next, the subdimension of transformational leadership is introduced into the second-layer model. The Durbin–Watson coefficient of multiple regression is 1.876, the tolerance is between 0 and 1, and the maximum value of the variance inflation factor VIF is 2.205. The regression model has no autocorrelation and common linearity. The dimensions entered into the regression model after stepwise analysis include intelligence stimulation and charisma influence. The model explained a total of 39.7% of teachers' teaching innovation, of which intelligence stimulation explained 36.7% of teachers' teaching innovation and charisma influence explained 1.5%. The joint prediction variance of the second-level regression model relative to the control variable increased by 0.011, indicating that the introduction of transformational leadership dimensions into the regression model increased the model's interpretation by 1.1%. From the perspective of standardized regression coefficients, the *β* coefficients of intelligence stimulation and charisma are 0.438 and 0.213, respectively. These two dimensions have a positive impact on teachers' teaching innovation, while other control variables have no significant impact on teachers' teaching innovation. Therefore, it can be concluded that both intellectual stimulation and charismatic influence in transformational leadership can promote teachers' teaching innovation, while vision stimulation and individualized care have no significant correlation with teaching innovation. The standardized regression equation can be expressed as teacher teaching innovation = 0.438 × intelligence stimulation + 0.213 × charisma influence.

### 4.5. Analysis of Results

Under the premise of controlling for demographic variables such as teacher gender, age, and teaching subject, this research uses transformational leadership as the explanatory variable, teacher teaching management as the explained variable, and the school's organizational innovation atmosphere as the mediating variable for regression analysis. The inspection yielded the following results. The transformational leadership of principals perceived by teachers has a significant predictive effect on teachers' teaching management, indicating that the practice of transformational leadership by principals is a necessary path to improve the teaching management level of school teachers. Its subdimension intelligence stimulation and charismatic influence also have a positive effect on teaching innovation, while vision stimulation and individualized care have no significant impact on teaching innovation, and the positive effects of transformational leadership should be properly used. Research hypotheses H1, H1a, and H1d are verified, but H1b and H1c cannot be verified. The details are shown in Table 6.

## 5. Conclusion

In the descriptive statistical analysis of this study, the transformational leadership style of college principals has a positive impact on teachers' teaching innovation. There is a positive correlation between charisma and teachers' teaching management, and there is a positive correlation between intellectual stimulation and teachers' teaching management. From the data, it can be concluded that the average score of individualized care in the subdimension of transformational leadership is much lower than the scores of other dimensions. And it reaches a statistically significant level, indicating that teachers' perceived leadership care and the work support is far from the expected level. To a certain extent, the principal's excessive alienation and weakening of communication with teachers is a true portrayal of the bureaucratic tendency of the current primary and secondary school organizations, which is not conducive to the effective development of teaching innovation activities. The score is much higher than other dimensions, indicating that the principal is actively exerting personal influence, prompting teachers to resonate with the school's collective mission, and at the same time fully publicizing their own personality charm and noble character, and stimulating teachers' worship and awe of themselves through various methods. Transformational leadership and its subdimension intelligence stimulation and charismatic influence can effectively predict teachers' innovative teaching levels; that is, the higher the principal's transformational leadership level, the stronger teachers' teaching innovation ability and the predictive effect of intelligence stimulation on teachers' teaching innovation. There are also some shortcomings in this study. For example, the influence of factors such as teachers' interpersonal relationships and organizational learning was not considered in the questionnaire design, and these factors were not controlled in the subsequent empirical analysis.

## Figures and Tables

**Figure 1:** Confirmatory factor analysis model.

**Table 1:** Transformational leadership style measurement items.

Transformational leadership style	Variable dimension	Measurement item
	Glamour influence	Sacrificing personal interests for the collective good
		Talk about important values and beliefs
		Emphasize the importance of a school's collective sense of mission
		Actively talk about what needs to be done
		Do not take the fruits of other people's labor as your own
		Allow teachers to understand the development prospects of the school
		Show power and confidence
	Vision incentive	Allow teachers to understand the school's development philosophy and development goals
		A promising future for everyone
		Explain the long-term significance of the work to the teacher
		Provide teachers with clear goals and directions
		Frequently work with teachers to analyze the impact of their work on the overall goals of the school
		Willingness to increase teacher effort
	Intellectual stimulation	Re-examine whether key assumptions are correct
		Always encourage teachers to use various methods to solve problems
		Often suggest new work, teaching methods to me
		Guide teachers to consider problems with new thinking and complete set tasks
		Old problems also require us to think differently
	Personalized care	In the process of dealing with teachers, the actual situation of teachers will be considered
		Frequent communication with teachers to understand teachers' work, life, and family situations
		Patiently teach teachers and answer questions for teachers
		See teachers as individuals, not just general members of the organization
		Focus on creating conditions for teachers to give full play to their strengths

**Table 2:** Reliability analysis of the questionnaire.

Variables and dimensions	Number of measurement items	Cronbach's alpha coefficient	Reliability level
Transformational leadership	17	0.975	Very high
Glamour influence	4	0.892	High
Vision incentive	4	0.929	Very high
Intellectual stimulation	5	0.932	Very high
Personalized care	4	0.942	Very high

**Table 3:** Evaluation indicators for the goodness of fit of the transformational leadership overall model.

Statistical test	*x* ^2^/d*f*	RMESA	RMR	TLI	GFI	CFI	IFI
Fit criteria	1–5	<0.08	<0.05	>0.90	>0.90	>0.90	>0.90
Inspection data	4.711	0.060	0.012	0.973	0.941	0.978	0.978

**Table 4:** Descriptive statistical analysis of transformational leadership.

Variables and dimensions	Average value	Standard deviation	Post hoc multiple comparisons (*P* < 0.05)
Transformational leadership	4.1686	0.63583	Charisma influence > vision inspiration > personalized care
Glamour influence	4.2554	0.58808	
Vision incentive	4.1580	0.69812	
Intellectual stimulation	4.1466	0.64921	
Personalized care	4.1201	0.76199	

**Table 5:** Transformational leadership and the impact of its dimensions on teacher teaching innovation.

Variable	Level one			Second floor			Multicollinearity test			
	Beta B	Sig Beta	B Sig	Beta B	Sig Beta	B Sig	Tol	VIF	Tol	VIF
Gender	−0.015	0.599	0.425	−0.014	−0.552	0.458	0.893	1.120	0.893	1.120
Teaching age	0.003	0.035	0.915	0.003	0.030	0.925	0.454	2.203	0.453	2.206
Education	0.020	0.809	0.359	0.024	0.941	0.282	0.674	1.483	0.674	1.484
School section	−0.010	−0.245	0.675	−0.004	−0.104	0.859	0.579	1.728	0.573	1.745
Job title	−0.054	−1.474	0.037	−0.050	−1.373	0.050	0.506	1.976	0.506	1.977
School	−0.024	−1.212	0.217	−0.024	−1.217	0.211	0.890	1.124	0.889	1.125
Subject	−0.003	−0.032	0.878	−0.004	−0.038	0.855	0.814	1.228	0.814	1.229
Change leadership	0.806	1.342	0.000				0.978	1.023		
Intellectual stimulation				0.388	2.154	0.000			0.130	7.680
Personal care				0.308	1.821	0.000			0.182	5.481
Vision incentive				0.143	0.920	0.003			0.144	6.937
*R*2	0.662			0.669			DW		1.748	
Δ*R*2	0.659			0.666					1.788	
*F*	247.862			204.520						

**Table 6:** Analysis of regression results.

Assumption	Hypothetical content	Validation results
H1	The transformational leadership style of college principals has a positive impact on teachers' teaching innovation	Support
H1a	There is a positive correlation between the influence of charm and teachers' teaching management	Support
H1b	There is a positive correlation between vision incentive and teacher teaching management	Does not support
H1c	There is a positive correlation between individualized care and teachers' teaching management	Does not support
H1d	There is a positive correlation between intellectual stimulation and teachers' teaching management	Support

## Data Availability

The dataset can be accessed upon request.
